# A Fact-Finding Procedure Integrating Machine Learning and AHP Technique to Predict Delayed Diagnosis of Bladder Patients with Hematuria

**DOI:** 10.1155/2021/3831453

**Published:** 2021-08-21

**Authors:** Chia-Lun Lo, Ya-Hui Yang, Hsiao-Ting Tseng

**Affiliations:** ^1^Department of Health-Business Administration, Fooyin University, Kaohsiung 83102, Taiwan; ^2^Department of Information Management, National Central University, Taoyuan 32001, Taiwan

## Abstract

Bladder cancer, the ninth most common cancer worldwide, requires fast diagnosis and treatment to prevent disease progression and improve patient survival. However, patients with bladder cancer often experience considerable delays in diagnosis. One reason for such delays is that hematuria, a major symptom of bladder cancer, has a high probability of also being a warning sign for urinary tract diseases. Another reason is that the sensitivity of the body parts affected by bladder cancer deters patients from undergoing cystoscopy and influences patients' “physician shopping” behavior. In this study, the analytic hierarchy process was used to determine critical variables influencing delayed diagnosis; moreover, the variables were used to construct models for predicting delayed diagnosis in patients with hematuria by using several machine learning techniques. Furthermore, the critical variables associated with delayed diagnosis of bladder cancer in patients with hematuria were evaluated using GainRatio technology. The study sample was selected from a population-based database. The model evaluation results indicated that the prediction model established using decision tree algorithms outperformed the other models. The critical risk factors for delayed diagnosis of bladder cancer were as follows: (1) cystoscopy performed 6 months after hematuria diagnosis and (2) physician shopping.

## 1. Introduction

Over the past 20 years, advances in technology and the popularization of social networks have facilitated the transmission of medical knowledge and information; this has enabled the public to acquire medical-related knowledge online and thus reduced medical information asymmetry [1]. Many patients actively seek additional medical opinions from multiple physicians to obtain more information on the medications or diagnoses they have obtained from the Internet. However, the increasing complexity of disease treatment strategies has increased the likelihood of physician misjudgment. According to a Harvard University study, 3.7% of hospitalized patients experienced medical injury, 27.6% experienced medical negligence, 69% experienced a human error, 2.6% experienced permanent disability, and 13.6% died due to medical errors [2]. Accordingly, reducing medical errors is a crucial issue in the medical field.

Most medical errors can be prevented, and the prevention of diagnostic delay can serve as a starting point to effectively reduce such errors [3–6]. Diagnostic delay not only causes poor prognosis but also increases medical expenses and affects quality of life. However, diagnostic delay is associated with the autonomy and professionalism of the physician; hence, this topic has rarely been explored. Several relevant medical studies have discussed major diseases that are difficult to diagnose, such as bladder cancer.

The incidence of bladder cancer has increased with urbanization and industrialization. Bladder cancer is the most common malignant neoplasm in the urinary system and the ninth most common cancer worldwide, causing more than 165,000 deaths each year [7]. The incidence of bladder cancer is three times higher among men than among women [8, 9]. The most notable symptom of bladder cancer, namely, hematuria, is not unique to the disease, causing difficulty in diagnosis. In addition, because bladder cancer has a 50%–70% chance of recurrence and a 30%–40% chance of increased malignancy after recurrence, accurate diagnosis without delay is crucial [9].

In general, the main symptom of bladder cancer is hematuria. Therefore, the primary method of diagnosing bladder cancer entails visually checking for hematuria symptoms or performing a urine test for detecting blood reactions or cancer cells [10]. This method is simple and fast. However, hematuria is caused by various factors, and situations with unknown causes also exist. Moreover, the fact that hematuria is a painless symptom, that early symptoms of bladder cancer may be unapparent, and that the condition can be overlooked by the patient may result in misdiagnosis.

Hematuria is often discovered inadvertently, but it has a high probability of being a warning sign for urinary tract diseases. Hematuria may be caused by numerous other factors, such as lithiasis, urinary tract infection, and malignant tumors. However, even if patients are detected to have hematuria, a timely follow-up examination and tracking may not be conducted because of numerous influencing factors. For example, patients with bladder cancer may not have visible hematuria symptoms. Even if patients discover the symptoms, they may visit the nephrology or gynecology department rather than the urology department. In particular, female patients may initially visit the gynecology department (gynecological diseases can also cause hematuria). Bladder cancer may not be considered a possibility by gynecologists, and the lack of immediate judgment and further tests leads to diagnostic delays. When cancer is finally detected, the treatment may have been delayed beyond the optimal time. Such misdiagnoses can cause considerable physical and mental harm to patients and their family members.

The secondary method of diagnosing bladder cancer is cystoscopy. However, the examination of sensitive body parts, requirement of anesthesia, and physical discomfort after examination may deter patients from undergoing cystoscopy, eventually causing diagnostic delays. Studies have highlighted that delays can be caused by numerous factors, including limited awareness of guidelines, variations in recommendations by different guidelines, low perceived yield of cystoscopy in patients with hematuria, urgency, poor communication within and between clinical teams, and failures in patient adherence to prescribed plans [11–18]. Therefore, satisfactory noninvasive examination methods for the early diagnosis and accurate and timely monitoring of recurrence of bladder cancer are unavailable. Diagnostic delay implies a physician's negligent behavior and disregard for relevant patient symptoms, which may cause harm to patients. Nevertheless, if patients exhibit different symptoms for the same disease, physicians face higher risks and pressure during diagnosis. Thus, a predictive tool to facilitate early diagnosis would be valuable for clinical physicians.

The possible influence of diagnostic delay on survival and the risk factors for diagnostic delay in patients with cancer have been subjects of considerable interest and controversy for several years. Clinicians have traditionally been concerned with cancer-related research; nevertheless, most patients (especially those with cancer) face an unexpected or ambiguous situation and are generally eager to seek a second opinion from another physician to confirm their initial diagnosis. Even in such circumstances, patients and their family members face difficulties in choosing a treatment method and are faced with the following questions: “Why me?” or “Is the diagnosis real?” or “Is there a better treatment strategy?” Lower compliance with physicians' orders and chaotic “physician shopping” behaviors leads to the possibility of delayed diagnosis [19]. However, establishing a systematic support method for patients' decision-making regarding treatment choices is difficult because patients have a complicated mindset that creates difficulties in decision-making; in addition, patients who do not make follow-up visits to consult the same physician are difficult to locate. Therefore, to address the problem of delayed diagnosis, determining how to track patients' physician shopping is crucial.

Accurately identifying patients' visiting conditions can be difficult, even in a single hospital. Accordingly, in this study, we first used the analytic hierarchy process (AHP) to investigate the criteria and priorities for delayed diagnosis of bladder cancer. We subsequently selected cases of hematuria with delays in bladder cancer diagnosis from Taiwan's nationwide population-based database established using information obtained from the National Health Insurance (NHI) system, which contains complete medical care visit information. Because this database is an observational database, its data reflect real-world medical care behavior patterns. Delayed diagnosis is a sensitive topic for clinicians; hence, it is not easily identified in practice. Consequently, establishing an accurate risk model for delayed diagnosis of bladder cancer remains challenging. To address this challenge, we used artificial intelligence (AI) methods to identify the factors causing diagnostic delays and establish prediction models for delayed diagnosis in patients with bladder cancer.

AI technology and its applications are prominent research areas. In recent years, an increasing number of AI applications have been introduced in the medical field. AI programs can perform clinical diagnostic procedures and recommend treatment suggestions. Numerous successful AI applications have been reported [20–29]. These applications use AI methods such as decision trees (DTs), support vector machines (SVMs), multilayer perceptron (MLP), and logistic regression (LGR). Moreover, these applications can help physicians in analyzing and understanding complex clinical data and help improve diagnosis and medical quality. Therefore, we used three types of AI methods—namely, decision tree-based classifiers (C4.5 and random forest), functional-based methods (SVM and logistic regression), and an integrated method (MLP)—to construct prediction models for delayed diagnosis and compared their performance in identifying delayed bladder cancer diagnosis. The following model performance measures were assessed in this study: accuracy, sensitivity, specificity, and area under the receiver operating characteristic curve (AUC).

## 2. Relevance of Bladder Cancer Review

Annually, more than 300,000 people are diagnosed as having bladder cancer worldwide. Bladder tumors rank as the seventh most common tumors and eighth most common cause of tumor-induced deaths. Bladder cancer is the most common malignant urinary tumors; 90% of the cases are transitional cell carcinoma, which renders early diagnosis difficult. Moreover, 5% of patients with bladder cancer develop metastasis by the time they are diagnosed. Bladder cancer typically occurs in people aged 50–70 years and is associated with the environment, smoking, and exposure to chemical substances. Studies have shown that 30%–50% of bladder cancers are caused by smoking and that smokers are 2–4 times more likely to develop bladder cancer compared with nonsmokers. Diagnosis and staging are performed through analysis of patients' medical history, urinalysis, cystoscopy, and urine cytology [8, 9].

Frequent urination, urgent urination, and pain during urination are initial symptoms of bladder cancer. The most common primary symptom in the early stage is hematuria, particularly manifested as repeated occurrence of blood in urine without pain during urination, which can be observed by either the naked eye or a microscope. Men and women should pay attention to the presence of blood in urine. Hematuria can be divided into initial, terminal, and total hematuria. However, hematuria is caused by various factors, such as urinary tract infection, urinary tract stones, urinary tract cancer, benign prostatic hyperplasia, kidney diseases, coagulation disorders, and medication; therefore, the diagnosis of bladder cancer is difficult [9, 10].

Bladder cancer is diagnosed using methods and tools such as routine urine tests, intravenous pyelography (IVP), ultrasound examination, urine cytology, and cystoscopy. However, IVP and ultrasound examination cannot detect small tumors or foreign bodies. The cell staining technique employed in urine cytology is Papanicolaou staining, which exhibits high specificity but is insensitive to urothelial carcinoma with low malignant potential, resulting in a high rate of false negative results. Therefore, in clinical practice, other tests are conducted in conjunction with this method. Alternatively, pathologists can determine the presence of cancer cells according to the cell types and characteristics. Even if the presence of a tumor is confirmed by X-ray and ultrasound tests, these tests cannot reveal whether the tumor is benign or malignant. Bladder cancer is not detected in the first test in many cases; this is either typical or because cancer cannot yet be detected using equipment. Therefore, patients with hematuria who are determined as exhibiting no bladder cancer in their tests are generally recommended to have a follow-up examination within 3–6 months. Nevertheless, in clinical practice, the cause of repeat hematuria in some patients cannot be identified [8, 9].

Therefore, cystoscopy is generally the primary means of examining bladder cancer in clinical practice. Cystoscopy is conducted to detect overall changes in the bladder, ureteral orifice, prostate gland, and urinary tract. Other symptoms in patients, such as difficulty urinating, narrowing of the prostate or urinary tract, or hematuria of unknown causes, can be examined through cystoscopy for further information. When the presence of a tumor is confirmed, its appearance and characteristics can be observed with the naked eye through cystoscopy. Subsequently, a biopsy can be performed to determine the stage of cancer and facilitate accurate diagnosis.

However, because cystoscopy is expensive and involves sensitive, invasive, and uncomfortable procedures, it is often avoided by patients and is usually not the first choice for physicians, resulting in delayed diagnosis of bladder cancer. Occasionally, physicians are misled by the self-reported symptoms of patients in their diagnostic decision-making. They occasionally use patients' vague self-reported symptoms as a clue for diagnosis; lack a holistic, systematic, or comprehensive analysis; or fail to consider a scientific basis as necessary for a diagnostic decision. These factors often lead to time delays and hence to delayed diagnosis.

## 3. Materials and Methods

### 3.1. Database and Ethical Consideration

For tracking patient physician shopping, population-based health data were used in this study. This case-control study used data retrieved from Taiwan's National Health Insurance Research Database (NHIRD) for the period of 2005–2013. Data in the NHIRD are derived from medical claims records of the Taiwan NHI program and include original medical claims and registration files for 1,000,000 enrollees of the NHI program. Taiwan's National Health Research Institutes randomly selected these 1,000,000 enrollees from all enrollees listed in the 2005 Registry of Beneficiaries (*n* = 23.72 million). The NHIRD is one of the largest and most comprehensive population-based datasets in the world. Previous studies have demonstrated the high validity of the data derived from the NHI program. In our empirical analysis, we used a large dataset sourced from Taiwan's NHIRD for the years 2005–2013.

The Institutional Review Board of Fooyin University Hospital approved this study (protocol number: FYH-IRB-106-06-06-02-A). Written consent from the study patients was not obtained because the NHIRD consists of deidentified secondary data for research purposes, and the Institutional Review Board of Fooyin University Hospital issued a formal written waiver regarding the need for consent.

### 3.2. Structure of the Decision-Making Model

To resolve the complications and confusing alternatives, the AHP was used to decide which input variable would be suitable for use in the models. The AHP is a research methodology developed by Thomas L. Saaty in 1971. It is mainly applied to uncertain situations and decision-making problems with multiple evaluation criteria [30]. The basic concept of AHP theory is the pairwise comparison derived from the mechanism of idea formation in the human brain. The human brain can easily make adequate judgments in a pairwise comparison but tends to become muddled in the case of multiple alternatives. In the AHP, the opinions of experts and decision-makers are collected, and through consistency verification, the experts' comparison results on each dimension are presented logically and coherently. A decision-making problem is decomposed into a hierarchical decision-making process, and each element that constitutes the hierarchy is compared in a pairwise manner to set the priority scale. The following steps are involved in the AHP: (1) define the problem and determine the goal and (2) construct the hierarchical structure. The top level of the construction hierarchy is the goal of the problem, the middle level is the criterion, and the bottom level is the alternative. Therefore, we used the AHP to systematize the research questions. Subsequently, we applied an AHP expert questionnaire to collect and analyze the opinions of various experts in order to determine the factors influencing physician shopping in patients and consequently resulting in delayed diagnosis. After the assessment, 10 influential factors identified by the experts were included in the models for predicting the possibility of delayed diagnosis of bladder cancer in patients with hematuria. According to the experts' opinions, age of the patient and physician, seniority of the physician, hospital level and location, physician shopping, and cystoscopy record within 6 months were possible influential factors.

In general, AHP structures for two decision steps are similar. The AHP structure in this study had three levels. The first level pertained to the delayed diagnosis of bladder cancer in patients with hematuria, the second level involved the classification of the criteria, and the third level involved the subcriteria. The consistency index for the criteria of the AHP structure was 0.084, and the random index (RI) was 1.49. Accordingly, the consistency ratio (CR) was calculated as 0.056. According to Saaty's suggestion, when the CR is ≤ 0.10, the matrix is consistent and the experts' opinions are acceptable. The ranks of the variables are presented in Table 1.

### 3.3. Study Population Selection and Controls

Regarding our study sample, we selected patients who were newly diagnosed as having hematuria (International Classification of Diseases, Ninth Revision, Clinical Modification (ICD9-CM) code 599.7) or blood in the stool (ICD9-CM code 578.1) between January 1, 2005, and December 31, 2013, in the NHIRD. For this retrospective case-control study, cases were included without any recruitment restrictions on age, sex, ethnicity, or cancer stage.

In the preprocessing stage, to identify patients with an actual diagnosis of a malignant neoplasm of the bladder, we selected those who were diagnosed twice as having a malignant neoplasm of the bladder (ICD9-CM code 188.9) from CD (i.e., “ambulatory care expenditures by visits”) files in the NHIRD. Thus, we identified 607 patients. Patients who were suspected to have a malignant neoplasm of the bladder were not included. In addition, two patients with unknown date of birth and without sex information and 58 patients without any cystoscopy record were excluded. Moreover, 14 patients with bleeding in the digestive tract (ICD9-CM code 578.1) were removed to avoid confusion and to maintain the quality of the samples. The final sample comprised 535 patients with consistent information. For each patient, data such as physician shopping (including visits to surgery, gynecology, nephrology, Chinese medicine, and gastroenterology departments), frequency of visit, age and sex of the patient and physician, and region and accreditation of the hospital visited were collected from the database as predictors to determine whether the diagnosis was delayed. The outcome variable was delayed diagnosis; patients who were diagnosed as having a malignant neoplasm of the bladder at least 3 months after hematuria was recorded were defined as having delayed diagnosis and were thus assigned to the delayed diagnosis group (*n* = 210); otherwise, they were defined as not having delayed diagnosis and were thus assigned to the nondelayed diagnosis group (*n* = 325). 41% of patients were operated or administered other aggressive treatment 3 months after diagnosis of bladder cancer and were considered as having delayed diagnosis. The sample selection process is shown in Figure 1.

### 3.4. Classification Techniques

After feature selection according to experts' opinions in the AHP and the data retrieval process, prediction models for delayed diagnosis of bladder cancer were established using maximum likelihood (ML) technology. We applied several well-known ML-based single classification techniques, namely, DT, SVM, logistic regression (LGR), and MLP neural network with backpropagation classifiers.

A DT algorithm applies classification and induction methods to generate a tree-like decision structure that is learned by the inductive method of the known examples of each class. A DT is a useful ML model; it can process complex data and is not affected by linear regression and interactions between independent variables. DT nodes consist of branches and leaves; the decision node indicates the test to be performed. To classify the input data, each DT node is a predicate, and each predicate can determine whether the variable is greater than, equal to, or less than a prespecified value. During data analysis, if the selected data variable belongs to categorical data, it is called a classification tree; if the selected data variable belongs to the continuous pattern, it is called a regression tree. Data classification using a DT algorithm is a two-step process. The first step involves a learning process, wherein the training data are analyzed by the DT algorithm to create a model that is presented as classification rules or a DT. The next step involves determining the accuracy of the classification rules or DT. If the accuracy is acceptable, rules can be reused to classify new data in the same scenario of the practical field [29]. C4.5 and random forest are the two most commonly used DT-based learning techniques. A DT is similar to the clinical decision-making process of a physician. After a DT is modelized, it can provide a suitable method for explaining the problem at the hand. Therefore, we selected a DT algorithm in this study.

Vanik's research team at the AT&T Laboratory developed the SVM algorithm [31], which is a controlled classification algorithm based on statistical learning techniques. It devises a computationally efficient method of learning to separate hyperplanes in a high-dimensional feature space based on statistical learning theory. The SVM algorithm first projects the training instances into a high-dimensional vector space and then determines the separating hyperplane exhibiting a maximal margin (i.e., the distance between the separating hyperplane and the closest sample). To reduce the generalization error of the classifier, the SVM algorithm determines an optimal hyperplane or a set of optimal hyperplanes (i.e., a hyperplane with a maximal margin) to separate training instances into two or more classes. This hyperplane is then used to determine the class label of unknown instances. The SVM algorithm can be divided into two types: linear and nonlinear. The operating principle of the SVM is based on the principle of predicting the most appropriate decision function that separates two classes in the most appropriate way to achieve the best classification effect. Its major function is to process the classification problems encountered during the data mining process. LGR is also a widely used statistical technique for forecasting the value of a binary or ordinal variable. LGR predicts the probability of occurrence of an event by fitting data into a logistic function, thereby allowing inputs with any values to be transformed and confined to a value between 0 and 1. Each regression coefficient represents the corresponding variable's degree of contribution. A positive regression coefficient increases the probability of the output, whereas a negative regression coefficient decreases the probability of the output. Both SVM and LGR algorithms are functional-based learning techniques [32].

MLP is a mathematical model that imitates the functionality of biological neural systems [33, 34]. It consists of an input layer, an output layer, and one or more hidden layers. Neurons are organized and fully connected between two adjacent layers, and the output layer is responsible for producing estimated outputs. Each layer receives inputs from the previous layer and converts them into a higher level of combinations by using combination and transfer functions. A high learning rate may result in achieving the minimum error quickly but may lead to an MLP model periodically fluctuating around the solution without being able to converge. However, a low learning rate may result in a local minimum or a long time to converge [35].

### 3.5. Performance Measures

In this study, WEKA 37.3, an open-source ML program, was used to establish DT (C4.5, RF), SVM, LGR, and MLP prediction models for classification. Because the predictive performance of classifiers can be considerably influenced by the parameter settings, the CV parameter selection metalearner module implemented in WEKA was used to optimize the predictive performance of the selected classifiers. The specific values of the various parameters were combined for each classifier; subsequently, the optimal parameter setting was automatically determined based on the best prediction results obtained using the validation strategy of our study. The specific parameter range and values selected for each classifier are listed in Table 2. Previous studies have reported that several classification algorithms implemented in conjunction with AdaBoost achieved higher classification accuracy than did individual base classifiers [36–39]. In the present study, Adaptive Boost (or AdaBoost in short), a prominent classifier ensemble, was employed to further enhance the predictive power of the classifiers [40].

Tenfold cross-validation was applied to evaluate the predictive performance of the classifiers. Tenfold cross-validation is a practical statistical method in which sample data are divided into smaller subsets. The idea is to randomly divide the sample into 10 nonoverlapping subsamples, with the categories in each subsample similar to the original sample. Nine subsamples were used for training to establish the models, and the remaining (one) subsample was used for testing. The same procedure was performed 10 times (for all 10 combinations). For performance evaluation, the final accuracy was obtained by comparing the number of incorrect results with the original number of entries. The predictive performance of each classifier was measured by evaluating the accuracy, sensitivity, specificity, and AUC.

The most used empirical measure, accuracy, does not distinguish between the number of correct labels of different classes:

TP, true positives: number of examples predicted positive that are actually positive
FP, false positives: number of examples predicted positive that are actually negative
TN, true negatives: number of examples predicted negative that are actually negative
FN, false negatives: number of examples predicted negative that are actually positive
Accuracy: it refers to the total number of records that are correctly classified by the classifier. The accuracy of a classifier is defined as the percentage of test set tuples that are correctly classified by the model [31].
  (1) $$\begin{array}{c} \mathrm{Accuracy}=\frac{\mathrm{TP+TN}}{\mathrm{TP+TN+FP+FN}}. \end{array}$$
Sensitivity: refers to the true positive rate that means the proportion of positive tuples that were correctly identified [31].
  (2) $$\begin{array}{c} \mathrm{Sensitivity}=\frac{\mathrm{TP}}{\mathrm{TP+FN}}. \end{array}$$
Specificity: refers to the rate at which a test or diagnostic method sets a correct (i.e., negative) diagnosis for a patient who is not ill [31].
  (3) $$\begin{array}{c} \mathrm{Specificity}=\frac{\mathrm{TN}}{\mathrm{FP+TN}}. \end{array}$$

In general, if the predictive accuracy of the proposed model is perfect, its AUC is nearly 1. If the AUC is between 0.8 and 0.9, then the model has high predictive accuracy. If its AUC is between 0.7 and 0.8, then the proposed model is acceptable. We compared the pros and cons of each prediction model according to accuracy, sensitivity, specificity, and AUC and then selected the most appropriate model for predicting the course of disease possible delay diagnosis of bladder cancer in patients with hematuria.

## 4. Results and Discussion

### 4.1. Patient Selection

Table 2 presents the variables and descriptive statistics of the delayed and nondelayed diagnosis groups. The delayed diagnosis group comprised 210 patients with bladder cancer, and the nondelayed diagnosis group had 325 patients, of whom 67%-68% were men. The median age at enrollment was approximately 67 years in both groups (interquartile ranges: 31–93 and 16–98 years). Physician shopping behaviors in both groups were for surgery, gynecology, Chinese medicine, gastroenterology, and nephrology. In the delayed diagnosis group, over 97% of the patients underwent cystoscopy after hematuria was detected after a delay of 6 months, which means that delayed cystoscopy caused significantly delayed diagnosis. The demographics of patients and physicians and other variables are presented in Table 3.

### 4.2. Experimental Results for Different Models

Next, we combined the two groups (i.e., patients and physicians) to establish prediction models of delayed diagnosed in order to assist physicians in identifying patients at a high risk of bladder cancer. According to the law of large numbers, some useful instances in the study data may not be chosen by the classifier; therefore, we applied the models 30 times to construct datasets (by seed = 1–30) and averaged the evaluation results. For each generated dataset, tenfold cross-validation was applied in all the experimental evaluations. To evaluate the performance of our model, parameters such as accuracy, sensitivity, specificity, and AUC were considered.

The evaluation results for the six classifiers (i.e., C4.5, RT, random forest, SVM, logistic regression, and MLP) in the prediction models are presented in Table 4. For ease of explanation, this table presents only the mean and standard deviation of the 30 generated datasets. Summaries of other statistics are available upon request from the authors.

First, the average predictive accuracy rates of the C4.5 and RT classifiers were 0.859 and 0.879. These classifiers outperformed the SVM (0.746), LGR (0.788), and MLP (0.742) classifiers. The average sensitivity levels of the C4.5, RT, SVM, LGR, and MLP classifiers were 0.843, 0.875, 0.752, 0.799, and 0.720, respectively; their specificity levels were 0.858, 0.872, 0.769, 0.802, and 0.709, respectively; and their average AUC values were 0.871, 0.942, 0.705, 0.854, and 0.775, respectively. Apart from the SVM classifier, all the classifiers exhibited excellent predictive performance because the AUC values were >0.7. The tree-based classifiers (i.e., C4.5 and RF) outperformed the functional-based classifiers (SVM and LGR) and MLP in terms of prediction accuracy. Moreover, the average sensitivity and specificity levels of the C4.5 and RF classifiers were higher than those of the SVM, LGR, and MLP classifiers. As expected, the DT-based classifiers outperformed the other classifiers in terms of the five selected performance indicators. Therefore, we can conclude that the predictive performance of the DT-based classifier was superior to that of the functional-based and MLP classifiers; in particular, the RF classifier yielded superior accuracy compared with the other classifiers, and the difference was statistically significant (*P* < 0.05).

Second, our comparative results revealed an improvement in prediction ability—measured using all performance indicators in Table 4—when the classifiers were supplemented by AdaBoost. For example, the average accuracy, sensitivity, specificity, and AUC of the C4.5, RF, and MLP classifiers supplemented with AdaBoost were higher than those observed when these classifiers were implemented without AdaBoost; nevertheless, the difference not statistically significant. However, the SVM classifier supplemented with AdaBoost exhibited relatively low performance in one of the indicators than it did when implemented without AdaBoost; this means that the predictive performance was not stable. The evaluation results for the LGR classifier revealed a similar trend.

### 4.3. Variable Important Evaluation

In addition to comparing the performance of the classifiers in determining delayed diagnosis of bladder cancer, we determined their predictive performance. We further evaluated the importance ranking of each selected variable of patients' physician shopping by using ML technology. The GainRatioAttributeEval model in WEKA was used to evaluate the importance level of all variables selected in this study. In the model, the gain ratio index was computed for each input variable; this index helped us in determining the relative importance of the variables.

As given in Table 5, we adjusted the input variables for our models (e.g., DT-based classifiers) for improving the model performance continually by calculating the gain ratios. We observed that hematuria was the most crucial variable influencing delayed diagnosis. However, undergoing cystoscopy 6 months after symptom appearance was determined to be the main reason for delayed diagnosis of bladder cancer, followed by variables related to patients' physician shopping. Many patients visit different departments to obtain more information about hematuria treatment strategies, contributing to a delayed diagnosis. Therefore, the mental stress associated with undergoing cystoscopy in patients with hematuria should be assessed, and patients should be encouraged to accept cystoscopy, which can help prevent the “physician shopping” behavior.

The ML classifiers' evaluation of the variables was compared with the experts' opinions about the variable ranking list in Table 1. The clinical experts believed that if a patient with some symptoms undergoes cystoscopy, the physician should ask the patient to stay in the hospital for further treatment. However, because patients in such situations increasingly pursue a second opinion, physicians should endeavor to reduce the possibility of delayed diagnosis. The characteristics of the patient and their physician shopping behavior are crucial variables, and follow-up action and related strategies should be emphasized.

Objective ML classifiers were used in this study to determine data-driven criteria for delayed diagnosis in order to reduce subjective bias in humans. The results revealed that clinical staff should pay more attention to patients' physician shopping behavior. Delayed diagnosis usually occurs when clinical staff passively wait for patients to visit clinics. Therefore, clinical staff should actively contact patients to improve their awareness about treatment strategies for their diseases.

## 5. Discussion

This study developed ML models for predicting delayed diagnosis of bladder cancer following hematuria symptoms. The anamnesis, full urine, and cystoscopy examinations of 591 patients who visited a urology clinic in Taiwan were collected from the NHIRD. Five AI analysis classifiers, namely, C4.5, RF, SVM, LGR, and MLP algorithms, which are frequently utilized in medical diagnosis systems, were used to create classification models based on the dataset. All models were tested using tenfold cross-validation, and their classification performance levels were compared and evaluated.

The results reveal that delayed diagnosis was related to sex, patients' physician shopping (whether patients had visited the gastroenterology department and the number of patients' visits to gynecology and gastroenterology departments), physician seniority, and whether cystoscopy was performed. These results supported the study hypotheses. However, information on the patients' physiological factors was not available in the data. Thus, although we identified a relationship between the patients' physician shopping and delayed diagnosis, we could not exclude the possibility of bias or presence of additional factors causing delayed diagnosis.

For any disease, the optimal strategy for reducing the chance of a poor patient prognosis is early diagnosis. A critical objective of preventive health care is to promote early diagnosis based on the standard procedure of checking the medical history and symptoms. However, malignant neoplasms of the bladder are in a rather sensitive area of the body, and examination is uncomfortable. In addition, the medical field currently contains numerous specialized fields. Consequently, patients may visit the wrong department when seeking medical treatment. Delayed diagnosis may be the result of a combination of all these factors. Therefore, to avoid delayed diagnosis and unnecessary medical expenditures, physicians from departments other than the urology department should consider the possibility of malignant neoplasms of the bladder when examining patients with hematuria.

To reduce delayed diagnosis, coordination and communication across departments of the healthcare system are essential. When first-line medical service providers doubt the existence of other possibilities in their patients' conditions, they must think from a comprehensive perspective to reduce misjudgments, which is difficult. However, because disease treatment strategies and comorbidities have become increasingly complex, relying only on physicians' decisions is insufficient.

In recent years, with the rise of AI, scholars and practitioners in the medical field have increasingly used big data to improve diagnostic accuracy. Numerous factors might be associated with a malignant neoplasm of the bladder. However, because of the sensitivity of the location of the neoplasm, the necessity of adopting an invasive procedure, and the pain and pressure a patient experiences during the procedure, patients commonly avoid active treatment. Therefore, this study analyzed patients' behaviors associated with consulting physicians to determine the risk of delayed diagnosis. The findings can help in improving the quality of diagnosis of malignant neoplasms of the bladder. In the future, psychological data could be introduced into hybrid AI algorithms to improve prediction accuracy.

## 6. Conclusions

The main symptom of malignant neoplasms of the bladder is hematuria. However, hematuria is caused by various factors. Patients with hematuria often visit a department other than the urology department, leading to delayed diagnosis. Psychological factors such as fear are also common causes of delayed examination and thus delayed diagnosis. Therefore, incorporating technology to identify factors related to the diagnosis of patients with malignant neoplasms of the bladder would be valuable. In this study, supervised ML classifiers were applied to establish prediction models for determining the behavioral characteristics of patients that could lead to delayed diagnosis in order to reduce the chance of delayed diagnosis.

This study has several limitations. The prediction models of delayed diagnosis were established using medical data from the NHIRD. However, because of the limitation related to the value-added data analysis of NHI expenditure application data, further analysis of patients' psychological factors was not possible. Moreover, because of the lack of socioeconomic data, the patients could not be grouped to analyze behavioral differences among socioeconomic clusters to identify possible indirect effects. Therefore, we could only assume that causal relationships existed between the factors analyzed and delayed diagnosis. Finally, the behavioral patterns of patients cannot be the main reference for making a diagnosis.

In summary, the problem of delayed diagnosis is sensitive, and the lack of discussion in previous studies is probably due to the pressure to avoid medical disputes. However, value-based payment is an increasingly common trend in healthcare insurance policy. The accuracy of medical diagnosis must be actively improved to maintain high medical treatment quality. Therefore, future studies can consider including more factors to establish models for predicting delayed diagnosis or consider integrating prediction algorithms into a computerized physician order entry system to create a practical clinical decision support system with warning functions.

## Figures and Tables

**Figure 1:** Flowchart showing derivation of the study sample.

**Table 1:** The importance of variable ranking by AHP.

Rank	Dimension
1	Characteristics of patients
2	Cystoscopy after hematuria record for half year
3	Characteristics of hospital
4	Visiting behavior
5	Characteristics of physicians

**Table 2:** Parameter setting in Weka.

Method	Parameters	Range	Value setting
C4.5	Confidence factor	0.1–0.5	0.25
	Minimum number of instances per leaf	2–20	20

Random forest	Number of trees	5–250	10
	Number of attributes to be used in random selection	2–8	4

Support vector machines	Kernel		PolyKernel

Multilayer perceptron	Number of hidden nodes	5–10	7
	Learning rate	0.1–0.6	0.3
	Momentum factor	0–0.9	0.2
	Maximum number of epochs	300–900	500

**Table 3:** Characteristics of bladder cancer patients with delay diagnosed and control subjects.

Variables	Value	Delay diagnosed group (*n* = 210)	Nondelayed diagnosed group (*n* = 325)
Age	Patient	67.3 (31–93)	67.4 (16–98)
	Physician	54.7 (47–63)	56 (43–63)

Seniority (physician)		11.7 (4–20)	13 (5–20
Gender (patient)^*∗*^	Male	142 (67.6)	227 (68.8)
	Female	68 (32.4)	98 (30.2)

Gender (physician)^*∗*^	Male	201 (95.7)	313 (96.3)
	Female	9(4)	12 (3.7)

Hospital level^*∗*^	Medical center	60 (28.6)	113 (34.8)
	Regional hospital	81 (38.6)	135 (41.5)
	District hospital	36 (17.1)	43 (13.2)
	Clinic	33 (15.7)	32 (10.5)

Visit behavior^*∗*^	Surgery	52 (24.7)	19 (5.8)
	Gynecology	38 (18.1)	13 (4)
	Chinese medicine	48 (22.3)	3 (0.9)
	Gastroenterology	61 (29.0)	6 (1.8)
	Nephrology	53 (25.2)	30 (9.2)

Cystoscopy after hematuria record for half year		205 (97.6)	120 (36.9)
Visit times	Surgery	1.69	0.03
	Gynecology	1.69	0.05
	Chinese medicine	1.73	0.01
	Gastroenterology	0	0.02
	Nephrology	0	0.18

Location (level of urbanization)^*∗*^			
	City	82 (39.0)	114 (44.3)
	Commuting zone	54 (25.7)	80 (24.6)
	Towns and semidense areas	10 (4.8)	12 (3.7)
	Rural areas	64 (30.5)	89 (27.4)

^*∗*^*n* (%), the others are *μ*(*σ*).

**Table 4:** Performance results of classifiers.

Classifier	Algorithms	Accuracy, *μ*/*σ*	Sensitivity, *μ*/*σ*	Specificity, *μ*/*σ*	AUC, *μ*/*σ*
Without AdaBoost	C4.5	0.859/0.014	0.843/0.003	0.858/0.016	0.871/0.042
	RF	0.879/0.071	0.875/0.045	0.8720.081	0.942/0.048
	SVM	0.746/0.007	0.752/0.005	0.769/0.040	0.705/0.008
	LGR	0.788/0.011	0.799/0.013	0.802/0.021	0.854/0.011
	MLP	0.742/0.079	0.720/0.048	0.709/0.127	0.775/0.104

With AdaBoost	C4.5	0.856/0.088	0.825/0.109	0.856/0.088	0.915/0.064
	RF	0.881/0.066	0.857/0.062	0.881/0.066	0.943/0.045
	SVM	0.743/0.011	0.722/0.008	0.743/0.001	0.762/0.010
	LGR	0.791/0.002	0.802/0.025	0.791/0.003	0.828/0.008
	MLP	0.751/0.088	0.791/0.029	0.752/0.087	0.786/0.111

**Table 5:** Variable importance ranking by GainRatioAttributeEval.

Rank	Variable	GainRatio
1	Cystoscopy after hematuria record for half year	0.3030443
2	Gastroenterology visiting times	0.122365
3	Gastroenterology visiting	0.122365
4	Chinese medicine visiting	0.103643
5	Chinese medicine visiting times	0.0636328
6	Surgery visiting times	0.073374
7	Gynecology visiting times	0.063343
8	Nephrology visiting times	0.035427
9	Hospital level	0.007911
10	Location	0.004625

## Data Availability

The data used to support the findings of this study are available from the corresponding author upon request.
